RETRACTED

# Circular Ribonucleic Acid circFTO Promotes Angiogenesis and Impairs Blood–Retinal Barrier *Via* Targeting the miR-128-3p/Thioredoxin Interacting Protein Axis in Diabetic Retinopathy

**DOI:** 10.3389/fmolb.2021.685466

**Published:** 2021-08-04

**Authors:** Jianjin Guo, Feng Xiao, Wei Ren, Yikun Zhu, Qiujing Du, Qian Li, Xing Li

**Affiliations:** ^1^ Department of Endocrinology and Metabolism, The Second Hospital of Shanxi Medical University, Taiyuan, China; ^2^ Department of Oncology, The Second Hospital of Shanxi Medical University, Taiyuan, China; ^3^ Department of Endocrinology and Metabolism, Shanxi Bethune Hospital, Shanxi Academy of Medical Sciences, Taiyuan, China; ^4^ Shanxi Medical University, Taiyuan, China; ^5^ Shanxi Medical University, Jinzhong, China

**Keywords:** circFTO, MiR-128-3p, TXNIP, diabetic retinopathy, molecular biology

## Abstract

**Background:** Increasing attention has been attracted by the role of circular RNAs (circRNAs) in ocular diseases. Previous study has revealed that circ_0005941 (also known as circFTO, an alpha-ketoglutarate–dependent dioxygenase) was upregulated in the vitreous humor of diabetic retinopathy (DR), while its underlying mechanism in DR remains unknown.

**Methods:** Retinal vascular endothelial cells (RVECs) treated with high glucose (HG) were used to establish the DR cell model. The *in vivo* assays were conducted using streptozotocin-induced diabetic mice. The circular structure and stability of circFTO were identified by Sanger sequencing and RNase R treatment. RT-qPCR analysis was used to detect the RNA expression. The levels of the mRNA-encoded protein thioredoxin-interacting protein (TXNIP) or angiogenesis-associated proteins (VEGFA, PDGF, and ANG2) and blood–retinal barrier (BRB)-related proteins (ZO-1, Occludin, and Claudin-5) were measured by Western blot. The viability of RVECs was measured using CCK-8 assays. The angiogenesis of RVECs was assessed using tube formation assays *in vitro*. Endothelial permeability assays were conducted to examine the function of the BRB. The binding between genes was explored using RNA pulldown and luciferase reporter assays.

**Results:** CircFTO was upregulated in HG-treated RVECs. CircFTO deficiency reversed the HG-induced increase in the viability and angiogenesis of RVECs and alleviated HG-mediated impairment of the BRB. MiR-128-3p bound with circFTO and was downregulated in HG-treated RVECs. TXNIP was a downstream target gene of miR-128-3p. TXNIP was highly expressed in the DR cell model. Rescue assays revealed that circFTO promoted angiogenesis and impaired the blood–retinal barrier by upregulating TXNIP. In the DR mouse model, circFTO silencing inhibited angiogenesis and promoted BRB recovery *in vivo*.

RETRACTED

**Conclusion:** CircFTO promotes angiogenesis and impairs the blood–retinal barrier *in vitro* and *in vivo* by binding with miR-128-3p to upregulate TXNIP in DR.

## Introduction

Diabetic retinopathy (DR) is a common diabetic complication leading to blindness in patients in developed countries (Congdon et al., 2003). Risk factors such as genetic background, hyperglycaemia, hypertension, dyslipidaemia, puberty, and pregnancy all contribute to DR progression (Cheung et al., 2010). The lesions within the retina are symbolic features of DR, with changes in retinal blood vessels and neovascularization (Forbes and Cooper, 2013). It is estimated that approximately 80% of diabetic patients with over 20 years’ duration of diabetes show signs of DR (Leasher et al., 2016). The number of DR patients reaches 150 million worldwide and may be doubled by 2025 (Gupta et al., 2013). However, treatment for DR is still unsatisfactory, and it is necessary to explore the underlying mechanism for the improvement of therapy.

Circular RNAs (circRNAs) refer to endogenous noncoding RNAs in a covalently closed circular structure commonly present in eukaryotes (Chen, 2020). CircRNAs have been reported to be implicated in the pathogenesis of diverse diseases (Li et al., 2018), including ocular diseases (Guo et al., 2019; Zhang et al., 2020). For example, circular RNA-ZNF532 knockdown suppresses the degeneration of retinal pericytes and vascular dysfunction induced by diabetes (Jiang et al., 2020). CircRNA cPWWP2A facilitates retinal vascular dysfunction *via* the upregulation of Angiopoietin 1, Occludin, and sirtuin 1 (Yan et al., 2020). CircRNA_0084043 enhances the oxidative stress and inflammation response in DR progression *via* the upregulation of transforming growth factor alpha (TGFA) (Li et al., 2020). In this study, the role of circ_0005941 (also known as circFTO, an alpha-ketoglutarate–dependent dioxygenase) in DR was investigated. Previous study has revealed that circ_0005941 was upregulated in the DR vitreous humor (He et al., 2020), while its underlying regulatory mechanisms remain unclear.

CircRNAs exert their functions *via* diverse mechanisms, including the competitive endogenous RNA (ceRNA) network, in which circRNAs act as molecular sponges for miRNAs to restrain the suppressive effect of microRNAs (miRNAs) on messenger RNAs (mRNAs) (Hansen et al., 2013; Tay et al., 2014). Many circRNAs act as ceRNAs in the progression of DR. For example, circCOL1A2 acts as a ceRNA for miR-29b to upregulate the expression of the vascular endothelial growth factor (VEGF), which promotes angiogenesis in DR (Zou et al., 2020). CircRNA DMNT3B alleviates DR vascular dysfunction by serving as a ceRNA for miR-20b-5p to upregulate the expression of the bone morphogenetic protein and activin membrane bound inhibitor (BAMBI) (Zhu et al., 2019). Circ_0041795 acts as a ceRNA for miR-646 to activate the expression of vascular endothelial growth factor C (VEGFC), which facilitates the injury of high glucose–treated ARPE 19 cells in DR (Sun and Kang, 2020).

RETRACTED

In the present study, we hypothesized that circFTO might function as a ceRNA in DR progression, and the regulatory mechanism of circFTO in DR was further investigated using both *in vivo* and *in vitro* assays. The findings might provide a theoretical basis for DR treatment.

## Materials and Methods

### Bioinformatic Analysis

The starBase website (http://starbase.sysu.edu.cn/) was used to predict the miRNAs interacting with circFTO under the screening condition of CLIP-Data >= 2 and Degradome-Data >= 2 (Li et al., 2014). The downstream target genes of miR-128-5p were also predicted using the starBase website, and the top ten targets were identified based on the number of supported AGO CLIP-seq experiments (Ago-Exp-Num).

### Cell Culture

Human retinal vascular endothelial cells (RVECs) provided by the BeNa Culture Collection (Beijing, China) were maintained in Dulbecco’s modified Eagle’s medium (DMEM; Gibco, Grand Island, NY, United States) with 10% fetal bovine serum (FBS; Corning, Midland, MI, United States) and 1/100 penicillin/streptomycin (Biochrom, Cambridge, United Kingdom) at 37°C in 5% CO_2_. To establish the DR cell model, RVECs were treated with 5.5 mM glucose for the control group, 5 mM glucose and 25 mM mannitol for an osmotic control, or 30 mM d-glucose for the high glucose (HG) group (Zhu et al., 2019).

### Cell Transfection

Specific short hairpin RNAs (shRNAs) against the Cand negative control (NC) were purchased from GenePharma (Shanghai, China). For TXNIP overexpression, pcDNA3.1/TXNIP (Invitrogen, Shanghai, China) was synthesized with an empty pcDNA3.1 vector as a negative control. MiR-128-3p mimics and NC mimics were obtained from GenePharma. The plasmids were transfected into RVECs using Lipofectamine 2000 (Invitrogen) 4 days after HG treatment. The transfection efficiency was detected by RT-qPCR after 48 h.

### Actinomycin D and RNase R Treatments

Total RNA (2 μg) was cultured with or without 3U μg^−1^RNase R (Epicentre, Madison, WI, United States) at 37°C for 30 min. Next, the RNA was purified using an RNeasy MinElute cleaning kit (Qiagen), and the expression of circFTO or linear FTO was detected by RT-qPCR.

To examine the stability of mRNA, 2 mg/ml of Actinomycin D (Sigma-Aldrich, Shanghai, China) was used to treat RVECs, with dimethyl sulfoxide (DMSO) treatment as the negative control. The RNA expression level in RVECs was detected at specific time points (4, 8, and 12 h).

RETRACTED

### Reverse Transcription Quantitative Polymerase Chain Reaction

TRIzol reagent (Sigma-Aldrich) was used to extract total RNAs from human RVECs. The GoScript Reverse Transcription System (Qiagen GmbH, Germany) was used for RNA transcription. RT-qPCR was performed using a Universal RT-PCR Kit for circFTO and TXNIP and a TaqMan MicroRNA Assay Kit for miR-128-3p. RNA expression was calculated using the 2^-∆∆Ct^ method with normalization to GAPDH and U6. The primer sequences were as follows:

circFTO:

Forward: 5′-TGG​CTG​AGG​CAG​TTT​TGG​TT-3′,

Reverse: 5′-GGCATTGAGATCATCACACCCT-3’;miR-128-3p:

Forward: 5′-TCA​CAG​TGA​ACC​GGT​CTC​TTT​C-3′,

Reverse: 5′-CTCTACAGCTATATTGCCAGCCAC-3’;TXNIP:

Forward: 5′-TGG​ATG​GCT​CTC​AAG​ACA​G-3′,

Reverse: 5′-GGGATCCACCTCAGTATAAGTC-3’;GAPDH:

Forward: 5′-GAT​CAT​CAG​CAA​TGC​CTC​C-3′,

Reverse: 5′-TCC​ACG​ATA​CCA​AAG​TTG​TC-3’;

U6:

Forward: 5′-GGA​TCA​ATA​CAG​AGC​AGA​TAA​GC-3′,

Reverse: 5′-CTT​TCT​GAA​TTT​GCG​TGC​C-3’;

#### Cell-Counting Kit-8 Assay

The transfected RVECs were cultured in the medium at 37°C overnight. After trypsinization, RVECs were suspended in the medium (Jiang et al., 2009). Next, cells were plated onto 96-well plates at the density of 1 × 10^3^ cells/well. To detect the viability of RVECs, 10 μL of CCK-8 solution (Dojindo, Kumamoto, Japan) was added to each well and incubated for 4 h. After 48 h, a microplate reader (Reagen, Shenzhen, China) was used to determine the optical density (OD) at a wavelength of 450 nm. All experiments were conducted in triplicate.

### Western Blot

RVECs or mouse retinal tissues were lysed with RIPA buffer (Sigma-Aldrich), and total proteins were collected. The protein concentration was identified using a Pierce™ BCA Protein Assay Kit (Thermo Fisher, Shanghai, China). Next, the proteins were loaded on 10% SDS-polyacrylamide gel electrophoresis and transferred onto PVDF membranes. Subsequently, 5% nonfat milk was used to block the membranes for 2 h at ambient temperature and cultured overnight with primary antibodies, including anti-VEGFA (#ab214424, 1/1,000), anti-PDGF (#ab203911, 1/1,000), anti-ANG2 (#ab8452, 1/500), anti-TXNIP (#ab188865, 1/1,000), anti–ZO-1 (#ab276131, 1/1,000), anti-Occludin (#ab167161, 1/1,000), anti–Claudin-5 (#ab131259, 1/1,000), and anti-GAPDH (#ab8245, 1/1,000). GAPDH was set as the loading control. All antibodies were purchased from Abcam (Cambridge, United Kingdom). Then the membranes were cultured with secondary antibody at room temperature for 1 h in the dark. An enhanced chemiluminescence kit (ECL kit, Pierce Biotechnology, Rockford, IL, United States) was used to visualize the target signals of proteins. The protein levels were analyzed using ImageJ software (NIH, Bethesda, MA, United States) and normalized to the loading control GAPDH.

RETRACTED

### Ribonucleic Acid Pulldown Assay

RNA pulldown assay was used to explore the interaction between circFTO and potential binding miRNAs (miR-128-3p, miR-216a-3p, and miR-3681-3p). RVECs were lysed using Pierce IP Lysis Buffer (Thermo Scientific). A biotin-labeled circFTO probe (100 pmol) and oligonucleotide probes were mixed with the RVEC lysates added with 50 µL of streptavidin magnetic beads (Thermo Scientific) at 25°C overnight. Next, the RNAs pulled down using the oligo probe and circFTO probes were purified, extracted using an RNeasy Mini Kit (Qiagen) and detected by RT-qPCR analysis. The biotin-labeled RNA circFTO probe and control probes were designed and synthesized by RiboBio (Guangzhou, China), and the sequences of used RNA and probes are provided in Table 1.

**TABLE 1:** Sequences of RNA and probes used for ribonucleic acid pulldown assay.

	Sequences
Oligo probe	ATA​AGT​AAT​TGA​TTA​TAA​CAA​CTG​AGA​TTC​TAT​ACG​CCC​CTT​TAC​GGA​CGA​TTT​GAT​ATA​GCG​AGG​CTT​TAG​TAT​CCT​TTC​TCG​GTT​CCC​TGT​CAT​CGA​CGC​AAT​TAT​ATA​AAG​TCG​CAT​GAG​GAA​GTG​GCA​GTT​TAT​GCC​CGG​TAG​TTA​TGA​ACA​AGT​ATT​CAC​TGA​CGA​CCT​TGT​TGG​ATC​TAG​CGA​TGG​GTT​AAT​GTA​TAT​AAA​AAA​CCC​TGA​CTG​TAT​TAC​TCG​TAT​GCG​TTT​GAC​TAT​GAA​TTG​GTG​GTG​TAT​CAC​TGG​TTC​CTC​GAA​GTT​TCT​TTT​GTC​TGT​ACT​TTA​CTA​TGT​CAA​ACT​CAC​AAG​GTG​CTT​CTG​GGT​CCT​CCT​CTT​TCT​AGT​GCT​GGT​TTT​TAT​CAA​TAT​GAA​TAA​TTG​GGT​ATC​GTT​TCA​CTA​CGG​TCA​GGA​TAG​TAT​TGG​ATA​CTT​GGT​TTT​ACG​TTA​CTC​GTG​TTG​CCA​CTT​TCT​TAT​CTG​TGG​CAT​CAA​GGC​GTG​CTA​TTA​GAG​TTT​TTA​TCG​CCC​CAA​TAC​GTT​CAA​CCT​AGG​AGA​GGT​AAT​GGC​TTG​TGC​CAC​AGA​ATG​GCT​CGC​GTT​AAA​GCC​AAA​AAG​TAT​ACG​TCT​TCT​TCT​CCT​TCG​GAC​GCG​CAC​ACT​TAA​CGG​GAT​TTA​TCA​CCT​TGT​ATC​GAC​TAA​TGA​AAC​GCG​TCC​TTG​ATA​GCA​CAT​AAT​TTA​GGT​CAA​CTT​AAT​TTA​GAA​TGT​TGC​CAA​TCT​CCT​AGA​TAA​GAA​AAT​GTC​TTC​CGC​TTG​TCT​ACC​TCT​AAT​TCT​TTC​GAC​AGT​TTA​TTA​GTC​TGT​CTA​GTT​TTT​CTC​GTT​TGA​TTT​ATG​GAA​CTT​CCG​ATA​TAT​TGA​CAG​GGG​TTC​TGT​TGT​GTA​ATT​TCC​ACG​CCG​TTA​CTG​CAA​AGC​CTT​TGA​CGG​TGT​TTT​AAT​GAT​GAC​TAT​TCG​ACT​CTT​TAT​AGA​TGA​AAT​TAC​AUG​AGG​AUU​ACC​CAU​GUC​GAT​AGT​TTA​TGA​TGT​TTG​AAT​TGT​TGG​TAA​AAT​AAT​CTT​AAA​CAG​CGC​ACT​TAC​TTC​TAC​CTT​ATT​TCT
circFTO probe	GCCCTGAAGAGGAAAGTGAGGATGACTCTCATCTCGAAGGCAGGGATCCT GATATTTGGCATGTTGGTTTTAAGATCTCATGGGACATAGAGACACCTGG TTTGGCGATACCCCTTCACCAAGGAGACTGCTATTTCATGCTTGGTAATC TTTGGAAAATCAAAATTATATTGAAACTCTAGTGTCTAAATTTAGATTAT AGGATTTATATTTTGAGTATGTCTTATGAAATAAACTTTTGGAGTATTTT ATATTAAGAGCGAAACTTCTTTATAAGAACATGTAACTAGGTTTTTCTTT TTTGAGATATTGCTGATTTTTTGAGATGGAGCTTCACTCTTGTTGCCCAG GCTGGAGTGCAGTGGCACAATCTCTGCTCATTGCCGTTTCCACCTCCTGG ATTCAAGCAATTCTCCTTCCTCAGCCTCCCAAGTAGCTGGGATTACAGGC ACACACCAACACACCCAGTTAATATTTTGTATTTTTAGTAGAGATGGGTT TCACCACGTTGGCCAAGCTGGTCTCAAACTCCTGACCTCAGGTGATCCAC CTGCCTCGGTCCCCCAAAGTGCTGAGATTTACAGGACCATGCCCGGCCCA ATTAAAAGTTGTTTTTCTTTTTATTCTACATAGATGCAGAGTTCCTCAAA TATGCTAAACAATTTTCTGGATTCTTTATCAGAGATATTAAATCATCCAA GTCAAATTATAACTTTAAAAAATACTTTCCTGTCCGTATTAGTTTTTAGT AGTGAGAGTTTTTTTTTTTTTTCTTCTAGTTTTGAATGTTGTTTCTTCTC AGGAACAGCTGACCTGACAATGGGGCCTTTCTCTCGACTTGTCATTTAGT TCTTTGGGAAGCACAUGAGGAUUACCCAUGUAGTTTCTCAGTTGTGGTTA GGCCAACTGAAGCTGTGGAGTTTGTGAGGCTTTGTTTTTTTCTTCTTTGCT
miR-128-3p	5′-GGTCAGTGAACCGGTC-3′ 5′-GTGCAGGGTCCGAGGT-3′
miR-216a-3p	5′-TAATCTCAGCTGGCAACT-3′ 5′-GGTGTCGTGGAGTCG-3′
miR-3681-3p	5′-CTCTGTGCAGGGCCAACT-3′ 5′-CCAGTAGTGGATGAAGCAC-3′

RETRACTED

### Luciferase Reporter Assay

The pmirGLO vectors (Promega, Madison, WI, United States) subcloned with fragments of circFTO or TXNIP 3′UTR sequences containing the binding site to miR-128-3p were used to construct circFTO-WT/Mut vectors or TXNIP-WT/Mut vectors and then transfected into RVECs with miR-128-3p mimics or NC mimics. After 48 h of transfection, the dual-luciferase assay system (Promega) was used to examine the luciferase activity of WT/Mut reporters.

### Tube Formation Assay

The tube formation assay was conducted in triplicate to detect the angiogenesis of RVECs. After being starved in the medium for 24 h, RVECs were seeded in precooled 96-well plates with 60 μL of Matrigel (BD Biosciences, San Jose, CA, United States) at a density of 1 × 10^3^ for 18 h of incubation in the medium. Finally, an inverted microscope (Nikon, Tokyo, Japan) was used to take images, and Image‐Pro Plus (version 6.0) was used to calculate the meshes and branch length in the tube formation.

### Hematoxylin and Eosin Staining

The mouse retinal tissues embedded in paraffin in 5-μm slices were cultured in hematoxylin for 5 min. Then eosin dye solution was used to stain the tissue samples for 3 min. A microscope was used to capture the images of HE staining.

### Xenograft Animal Experiment

The animal experiment was approved by the ethical committee of The Second Hospital of Shanxi Medical University. A total of 32 C57Bl/6J male mice (5 weeks; weighing 20–25 g) were provided by Beijing Vital River Laboratory Animal Technology. The animals were randomly divided into the sham, DR, DR + AAV-empty, and DR + AAV-sh-circFTO groups (*n* = 8 per group). The mice were kept in a 12-h light/dark cycle with access to food and water. A DR mouse model was established by daily intraperitoneal injection of streptozotocin (STZ, 60 mg/kg, Sigma) into the mice successively for 5 days after the injection (IP) of ketamine (80 mg/kg) and xylazine (4 mg/kg) for anesthetization. Mice in the sham group were injected with an equal volume of citrate buffer. The fasting blood glucose of mice was accessed once a week. The diabetes was identified as successfully achieved when the fasting blood glucose of mice was over 300 mg/dl (Zou et al., 2020). Approximately 1.5 μL (1 × 10^12^ vg/mL) of adeno-associated virus (AAV)-5 with sh-circFTO or an empty vector was delivered into the vitreous humor using a 33-gauge needle two weeks before the diabetes induction (Shan et al., 2017). AAV5 was reported to effectively infect vascular endothelial cells and retinal pigment epithelial cells in previous studies, and recombinant AAV5 can be used to infect human retinal microvascular endothelial cells for gene expression depletion (Wu et al., 2017).

RETRACTED

### Blood–Retinal Barrier Breakdown Quantitation

Evans blue was employed to measure BRB breakdown, according to a previous study (Hossain et al., 2016). After the mice were anesthetized, Evans blue (45 mg/kg) was injected into them through the tail vein. 2 h later, the mice were re-anesthetized and blood samples (0.1–0.2 ml) were collected, and then the mice were euthanized. Next, the eyes were enucleated to dissect out the retina. Dimethylformamide treatment, centrifugation for retinas and blood samples, and the calculation of BRB breakdown were performed according to the previous study (Hossain et al., 2016).

### Statistical Analysis

All experiments were repeated three times, and data are shown as the mean ± standard deviation. The data were evaluated using SPSS 17.0 (IBM, Armonk, NY, United States). The differences between two groups were analyzed using Student’s *t*-test. The comparison among multiple groups was analyzed using one-way analysis of variance followed by Tukey’s *post hoc* analysis. The value of *p*< 0.05 was regarded as the threshold value.

## Results

### CircFTO Forms Closed Stable Circular Structure

The formation of circFTO is presented in Figure 1A. CircFTO comprising three exons at a length of 344 nucleotides was back-spliced by FTO premRNA. The splice junction that formed the circular structure of circFTO was confirmed by Sanger sequencing (Figure 1B). According to agarose gel electrophoresis (AGE) assay, circFTO was amplified only from cDNA with divergent primers, rather than in the products from genomic DNA, and FTO was amplified in both cDNA and gDNA (Figure 1C). As shown in Figure 1D, circFTO was more resistant to RNase R digestion than FTO. After Actinomycin D treatment, RT-qPCR showed that the half-life of circFTO was over 24 h, while that of FTO mRNA was approximately 14 h (Figure 1E).

RETRACTED

**FIGURE 1:** Stable circular structure of circFTO. **(A)** Formation of the circular structure of circFTO from FTO premRNA was schematically illustrated. **(B)** Sanger sequencing showed the splice junction of circFTO. **(C–E)** Agarose gel electrophoresis (AGE) and RNase R/Actinomycin D treatment were used to examine the circular structure of circFTO. **p<0.01, ***p<0.001.

### CircFTO Knockdown Alleviates High Glucose–Induced Angiogenesis and Blood–Retinal Barrier Breakdown in Retinal Vascular Endothelial Cells

According to RT-qPCR analysis, the expression of circFTO was significantly upregulated in RVECs treated with HG compared with that in the control and Mannitol groups (Figure 2A). The silencing efficiency of circFTO in HG-treated RVECs was confirmed using RT-qPCR analysis, showing that circFTO expression was markedly decreased in RVECs after HG treatment (Figure 2B). The viability of RVECs was increased in the group receiving HG treatment, while circFTO knockdown reversed the increase induced by HG treatment (Figure 2C). The RVEC angiogenesis was enhanced by HG treatment, while circFTO silencing decreased the number of meshes and the branch length in tube formation in RVECs after HG treatment (Figure 2D). Western blot analysis was used to detect the levels of angiogenesis-related proteins in RVECs. The protein levels of VEGFA, PDGF, and ANG2 were elevated in the HG group and showed a decrease in the HG+ sh-circFTO group compared with the HG group (Figure 2E). The levels of proteins (ZO-1, Occludin, and Claudin-5) associated with the blood–retinal barrier (BRB) were reduced in HG-treated RVECs, which was reversed by circFTO deficiency (Figure 2F).

**FIGURE 2:** CircFTO knockdown alleviates HG-induced angiogenesis and blood–retinal barrier (BRB) breakdown in RVECs. **(A)** RT-qPCR analysis was used to detect the expression of circFTO in RVECs treated with HG (30 mM glucose) or Mannitol (20 mM). **(B)** Silencing efficiency of circFTO in HG-treated RVECs was examined using RT-qPCR analysis. **(C)** RVEC viability in the control, Mannitol, HG, and HG+ sh-circFTO groups was detected using CCK-8 assays. **(D)** Angiogenesis of RVECs was assessed using tube formation assays after the indicated treatment. **(E)** Western blot analysis was used to detect the levels of angiogenesis-related proteins (VEGFA, PDGF, and ANG2) in RVECs. **(F)** Levels of proteins (ZO-1, Occludin, and Claudin-5) associated with the blood–retinal barrier (BRB) were measured by Western blot in RVECs in indicated groups. **p<0.01, ***p<0.001, &< 0.05, &&< 0.01, &&& < 0.001.

RETRACTED

### CircFTO Interacts With miR-128-3p in Retinal Vascular Endothelial Cells

As shown by the Venn diagram in Figure 3A, three miRNAs with a potential binding site to circFTO were predicted using the starBase website under the condition of CLIP >=2 and Degradome >=2. The results of RNA pulldown assay revealed that only miR-128-3p was significantly enriched in the circFTO probe, compared with the other candidate miRNAs (Figure 3B). Thus, miR-128-3p was selected for further study. The expression of miR-128-3p in RVECs treated with HG or Mannitol was detected using RT-qPCR. The results indicated that miR-128-3p was expressed at a low level in HG-treated RVECs (Figure 3C). Afterward, the overexpression efficiency of miR-128-3p was confirmed by RT-qPCR after the transfection of miR-128-3p mimics in RVECs (Figure 3D). The binding site between miR-128-3p and circFTO was presented. The results of luciferase reporter assay showed that miR-128-3p overexpression decreased the luciferase activity of wild-type circFTO in RVECs, while that of the mutant circFTO exhibited no significant change (Figure 3E). Moreover, the effect of circFTO knockdown on miR-128-3p expression was detected by RT-qPCR, showing that miR-128-3p expression was markedly upregulated due to circFTO deficiency (Figure 3F).

**FIGURE 3:** CircFTO interacts with miR-128-3p in RVECs. **(A)** Candidate miRNAs with a potential binding site to circFTO were selected using a Venn diagram under the condition of CLIP >=2 and Degradome >=2. **(B)** RNA pulldown assay was used to investigate the interaction between miR-128-3p and circFTO in RVECs using an oligo probe and a circFTO probe. **(C)** Expression of miR-128-3p in RVECs treated with HG or Mannitol was measured by RT-qPCR. **(D)** Overexpression efficiency of miR-128-3p in RVECs transfected with miR-128-3p mimics was examined using RT-qPCR. **(E)** Binding site between miR-128-3p and circFTO was predicted using the starBase website. A luciferase reporter assay was used to explore the binding between miR-128-3p and circFTO in RVECs transfected with miR-128-3p mimics. **(F)** RT-qPCR was performed to examine the effect of circFTO deficiency on the expression of miR-128-3p in RVECs. ***p<0.001.

### Thioredoxin-Interacting Protein Is Directly Targeted by miR-128-3p in Retinal Vascular Endothelial Cells

The expression of candidate mRNAs for miR-128-3p in RVECs transfected with miR-128-3p mimics was detected using RT-qPCR. The results showed that only TXNIP was significantly downregulated by miR-128-3p overexpression in RVECs (Figure 4A). Therefore, TXNIP was identified for further study. The protein level of TXNIP was also decreased after the transfection of miR-128-3p mimics in RVECs (Figure 4B). The mRNA expression and protein levels of TXNIP were all downregulated due to circFTO depletion, as shown by RT-qPCR and Western blot analyses (Figures 4C,D). Luciferase reporter assays demonstrated that miR-128-3p overexpression reduced the luciferase activity of Wt-TXNIP, and no evident change was observed in the TXNIP-Mut group (Figures 4E,F). RT-qPCR showed that TXNIP expression was elevated in RVECs treated with HG compared with that in the Mannitol or control group (Figure 4G).

RETRACTED

**FIGURE 4:** TXNIP is directly targeted by miR-128-3p in RVECs. **(A)** RT-qPCR was used to detect the expression of candidate mRNAs possessing binding sites with miR-128-3p in RVECs transfected with miR-128-3p mimics. **(B)** Western blot was used to measure the TXNIP protein level in RVECs with the transfection of miR-128-3p mimics. **(C)** mRNA expression of TXNIP was markedly decreased by silencing circFTO in RVECs, as shown by RT-qPCR. **(D)** Western blot analysis was conducted to detect the effect of circFTO knockdown on the protein level of TXNIP in RVECs. **(E,F)** Luciferase reporter assay was used to explore the relationship between miR-128-3p and TXNIP in RVECs. **(G)** RT-qPCR was used to detect TXNIP expression in RVECs in the control, Mannitol, and HG groups. **p<0.01, ***p<0.001.

### CircFTO Promotes Angiogenesis and Impairs the Blood–Retinal Barrier in Retinal Vascular Endothelial Cells by Upregulating Thioredoxin-Interacting Protein

The overexpression efficiency of TXNIP was verified in HG-treated RVECs. RT-qPCR revealed that TXNIP expression was successfully upregulated by pcDNA3.1/TXNIP (Figure 5A). Cell-counting kit-8 (CCK-8) assays revealed that TXNIP overexpression reduced the suppressive effect of circFTO silencing on the viability of RVECs (Figure 5B). The results of tube formation assay indicated that RVEC angiogenesis was inhibited by circFTO knockdown, while overexpressed TXNIP reversed the suppressive effect of silenced circFTO on RVEC angiogenesis (Figure 5C). Moreover, circFTO deficiency caused a reduction in the levels of angiogenesis-related proteins (VEGFA, PDGF, and ANG2), which was rescued by overexpressed TXNIP (Figure 5D). The levels of BRB-associated proteins (ZO-1, Occludin, and Claudin-5) were elevated after circFTO silencing and then reversed by TXNIP overexpression in RVECs (Figure 5E).

**FIGURE 5:** CircFTO promotes angiogenesis and impairs the blood–retinal barrier (BRB) in RVECs by upregulating TXNIP. **(A)** Overexpression efficiency of TXNIP in HG-treated RVECs was examined using RT-qPCR. **(B)** Viability of HG-treated RVECs after the transfection of sh-NC, sh-CircFTO, and sh-circFTO + TXNIP was detected by RT-qPCR. **(C)** Tube formation assay was used to assess the angiogenesis of HG-treated RVECs after the above transfection. **(D,E)** Western blot analyses were used to measure the levels of angiogenesis-related proteins (VEGFA, PDGF, and ANG2) and proteins associated with the BRB (ZO-1, Occludin, and Claudin-5) in HG-treated RVECs after the above transfection. **p<0.01, ***p<0.001, #< 0.05, ##< 0.01.

RETRACTED

### CircFTO Knockdown Attenuates Angiogenesis and Alleviates Blood–Retinal Barrier Breakdown Mediated by Diabetes in Diabetic Retinopathy Mouse Models

As shown by HE staining, in the DR mouse model (*n* = 8 mice/group), the mouse retinal cells were irregularly and disorderly arranged, and the number of vessels was increased. CircFTO deficiency attenuated these performances and alleviated the angiogenesis (Figure 6A). The thickness of the retina in mice was increased by DR, while circFTO deficiency partially reversed the DR-mediated increase in retinal thickness (Figure 6B). The breakdown of the BRB was measured using Evans blue dye, indicating that silencing circFTO mitigated the impairment of the BRB (Figure 6C). According to Western blot, the levels of angiogenesis-related proteins (VEGFA, PDGF, and ANG2) were elevated in DR mouse retinal tissues and then reversed by silenced circFTO. The levels of proteins associated with the BRB (ZO-1, Occludin, and Claudin-5) were reduced in DR mouse retinal tissues, and circFTO knockdown rescued the decrease in these protein levels (Figures 6D,E). RT-qPCR showed that circFTO and TXNIP expression levels were upregulated in DR mouse retinal tissues and decreased after circFTO knockdown, while the expression of miR-128-3p was downregulated in the DR mouse retinal tissues (*n* = 10) and showed an increase after the transfection of sh-circFTO (Figure 6F). Moreover, miR-128-3p expression was demonstrated to be negatively correlated with circFTO and TXNIP expression, while TXNIP expression was positively correlated with circFTO expression in mouse retinal tissues (n = 30), as identified using Spearman’s correlation coefficient (Figure 6G).

**FIGURE 6:** CircFTO knockdown attenuates angiogenesis and blood–retinal barrier (BRB) breakdown induced by diabetes in the DR mouse models. **(A)** HE staining showed the morphology of mouse retinal tissues in the sham, DR, DR + AAV-empty, and DR + AAV-sh-circFTO groups (*n* = 8 mice/group). **(B)** Thickness of the retina was quantified. **(C)** Breakdown of the BRB *in vivo* was measured using Evans blue. **(D,E)** Western blot analyses were used to detect the levels of angiogenesis-related proteins (VEGFA, PDGF, and ANG2) and proteins associated with the BRB (ZO-1, Occludin, and Claudin-5) in mouse retinal tissues in the above indicated groups. **(F)** Expression levels of circFTO, miR-128-3p, and TXNIP in mouse retinal tissues (*n* = 10) in the sham, DR, DR + AAV-empty, and DR + AAV-sh-circFTO groups were examined by RT-qPCR. **(G)** Expression correlation between every two genes of circFTO, miR-128-3p, and TXNIP in mouse retinal tissues (*n* = 30) was identified by Spearman’s correlation coefficient analysis. *p<0.05, **p<0.01, ***p<0.001.

RETRACTED

## Discussion

In the present study, circFTO was identified to be highly expressed in HG-treated RVECs. The knockdown of circFTO was revealed to reverse the HG-induced increase in the viability and angiogenesis of RVECs and alleviate the HG-induced impairment of the blood–retinal barrier (BRB). *In vivo* assays showed that circFTO silencing attenuated the angiogenesis and the impairment of the blood–retinal barrier induced by diabetes in the DR mouse models.

CircFTO was demonstrated to function as a ceRNA in the progression of DR. MiR-128-3p was revealed to be sponged by circFTO in RVECs and was demonstrated to be downregulated in HG-treated RVECs. The role of miR-128-3p has been reported in diverse diseases. For example, miR-128-3p is targeted by mmu_circ_0000250, which promotes the wound healing of diabetic mice (Shi et al., 2020). Moreover, previous studies have also indicated the aberrant expression profile of miR-128 in diabetic patients and diet-induced diabetic mice (Prabu et al., 2015). MiR-128-3p overexpression is revealed to promote inflammatory responses induced by TNF-alpha *via* regulating Sirt1 in bone marrow mesenchymal stem cells (Wu et al., 2020).

Thioredoxin-interacting protein (TXNIP) was revealed to be directly targeted by miR-128-3p at the 3′-untranslated region (3′-UTR) in RVECs. The expression of TXNIP at the mRNA and protein levels was negatively regulated by miR-128-3p and positively regulated by circFTO in RVECs. TXNIP was also upregulated in RVECs after HG treatment. Rescue assays indicated that TXNIP overexpression offset the effects of circFTO silencing on the viability, angiogenesis, and BRB of HG-treated RVECs. Previous studies have also reported that TXNIP was highly expressed in diabetic complications (Xu et al., 2013; Lv et al., 2020). For example, the inhibition of the p38/TXNIP/NF-κB pathway by melatonin is suggested to maintain the inner blood–retinal barrier in DR (Tang et al., 2021). Moreover, TXNIP overexpression has been demonstrated to activate autophagy and apoptosis in the rat müller cells treated with high glucose in DR (Ao et al., 2021). TXNIP deficiency is revealed to inhibit the NLRP3 axis and reduce renal damage in diabetic nephropathy rat models (Ke et al., 2020).

RETRACTED

In the progression of diabetes, retinal vessels are the early and common targets whose injury and dysfunction becomes a leading cause for vision loss in diabetic patients. The pathological alterations in the retina of diabetic patients are characterized by neovascularization (Nawaz et al., 2019). Molecules including vascular endothelial growth factor A (VEGFA), platelet-derived growth factor (PDGF), and angiogenin, ribonuclease A family, member 2 (ANG2) are closely related to angiogenesis, which increase vascular leakage and facilitate DR progression (Rask-Madsen and King, 2013). In this study, the expression levels of VEGFA, PDGF, and ANG2 were elevated after HG treatment, while circFTO silencing exerted a suppressive effect on the levels of these factors in HG-treated EVECs or the DR mouse model.

The blood–retinal barrier (BRB) is essential for the establishment and maintaining of a stable environment for optimum retinal function (Cunha-Vaz et al., 2011; Naylor et al., 2019), which is critically implicated in DR progression (Antonetti et al., 2021). The inner blood–retinal barrier (iBRB) comprises tight junctions (TJs) between neighboring retinal endothelial cells. As the first transmembrane protein that was identified in the TJ, Occuludin plays a vital role in paracellular permeability. Zonula occludens-1 (ZO-1) is a cytoplasmic protein that anchors transmembrane proteins to the cytoskeleton, which is important in the formation and organization of TJs (Bazzoni and Dejana, 2004; Naylor et al., 2019). Claudin-5 is the most predominant Claudin of the iBRB, which is confined to endothelial cells (Naylor et al., 2019). Herein, protein levels of ZO-1, Occuludin, and Claudin-5 were examined to probe the impairment of the BRB. When the BRB is broken down, protein levels of ZO-1, Occuludin, and Claudin-5 are downregulated. CircFTO promotes BRB breakdown by upregulating the expression of TXNIP in HG-induced RVECs and DR mouse models. Mechanistically, the mTOR inhibitor was reported to suppress the breakdown of the BRB, and mTOR signaling involved in pericytes might be profoundly relevant to early subclinical stages of DR (Jacot and Sherris, 2011). Despite the role of the mTOR pathway in DR, mTOR signaling is associated with the pathobiology of the retina. For example, the suppression of mTOR signaling inhibits the dedifferentiation of the retinal pigment epithelium, which is a critical factor involved in the formation of the outer blood–retinal barrier (Zhao et al., 2011). The association between mTOR and the regulation of TJs will be investigated in our future studies.

In conclusion, circFTO is upregulated in HG-treated RVECs, and circFTO promotes angiogenesis and impairs the BRB in HG-treated RVECs and in DR mouse models *in vitro* and *in vivo*, which might provide novel insight into DR treatment. However, more experiments are required in our future studies to further verify the upstream genes or downstream signaling pathways of the circFTO/miR-128-3p/TXNIP axis in DR development.

RETRACTED

## Data Availability

The original contributions presented in the study are included in the article/Supplementary Material; further inquiries can be directed to the corresponding author.
